RETRACTED

# The gastro protective effects of *Cibotium barometz* hair on ethanol-induced gastric ulcer in Sprague-Dawley rats

**DOI:** 10.1186/s12917-017-0949-z

**Published:** 2017-01-19

**Authors:** Nahla Saeed AL-Wajeeh, Maryam Hajerezaie, Suzita Mohd Noor, Mohammed Farouq Halabi, Nawal Al-Henhena, Ainnul Hamidah Syahadah Azizan, Sareh Kamran, Pouya Hassandarvish, Abdrabuh N. Shwter, Hamed karimian, Hapipah Mohd Ali, Mahmood Ameen Abdulla

**Affiliations:** 1 Department of Biomedical Science, Faculty of Medicine, University of Malaya, 50603 Kuala Lumpur, Malaysia; 2 Department of Microbiology, Faculty of Medicine, University of Malaya, 50603 Kuala Lumpur, Malaysia; 3 Department of Chemistry, Faculty of Science, University of Malaya, 50603 Kuala Lumpur, Malaysia

## Abstract

**Background:**

*Cibotium barometz* is a medical herb used traditionally in the Malaysian peninsula for several ailments, including gastric ulcer. The aim of this study was assessment the anti-ulcer effects of *C. barometz* hair on ethanol-induced stomach hemorrhagic abrasions in animals. Seven groups of Sprague Dawley (SD) rats were administered 10% Tween 20 in the normal control and ulcer control groups, and omeprazole 20 mg/kg and 62.5, 125, 250, and 500 mg/kg of *C. barometz* hair extract in the experimental groups. After 60 min, the normal control group of rats was orally administered 10% Tween 20, while absolute ethanol was orally administered to the groups of ulcer control, omeprazole and experimental groups. Stomachs of the rats were examined macroscopically and histologically. Homogenates of stomachs were used to evaluate endogenous antioxidant enzyme activities.

**Results:**

Rats pre-fed with plant extract presented a significant decrease in the sore area, increased pH of gastric contents and preserved stomach wall mucus compared to the ulcer group. Histologically, rats pre-fed with *C. barometz* hair extract showed mild to moderate disruptions of the surface epithelium while animals pre-fed with absolute ethanol showed severe disruptions of the stomach epithelium with edema and leucocyte penetration of the submucosal layer. A Periodic acid Schiff (PAS) staining revealed that each rat pre-treated with the plant extract displayed an intense uptake of stomach epithelial glycoprotein magenta color compared to the ulcer control group. Immunohistochemical analysis revealed that rats pre-fed with the plant extract showed an up-regulation of the heat shock protein 70 (HSP70) and down-regulation of Bax proteins compared to ulcer control rats. Homogenates of the stomach tissue demonstrated significant increases in the endogenous antioxidant enzymatic activity and decreased lipid peroxidation (MDA) in rats pre-treated with *C. barometz* hair extract compared with the ulcer control rats. In acute toxicity, the liver and kidney revealed no hepatotoxic or nephrotoxic effects histologically.

RETRACTED

**Conclusions:**

The gastric cytoprotective action of *C. barometz* hair extract might be attributed to antioxidants, an increase in gastric pH, stomach mucus preservation, increased endogenous antioxidant enzymes, decreased lipid peroxidation, up-regulation of HSP70 and down-regulation of Bax proteins.

## Background

Stomach ulcers are the common gastrointestinal and global disorders [1]. It occurs mainly due to the imbalance between the destructive and offensive factors of the mucosal barrier [2]. The destructive factors include stomach hydrochloric acid (HCl), mucosal hypoperfusion, free oxygen radicals, ethanol, *Helicobacter pylori* and excessive ingestion of non-steroidal anti-inflammatory drugs (NSAIDs) that promote the gastric mucosal injury and contribute to gastric ulceration [3].

The prevention or treatment of gastric ulcers is a medical challenge [4]. Gastric ulcer therapy has major disadvantages, including limited efficacy of drugs against the gastric illness and severe side effects [5]. Therefore, medicinal plants may be a viable alternative therapy that has fewer side effects and contains a wide variety of antioxidants. Medicinal plants are also promising alternative medications for the development of new drugs to control gastrointestinal diseases, which has been reviewed extensively in the literature [2, 6–12].

*Cibotium barometz* hair (family Dicksoniaceae) is known traditionally as “golden hair dog fern”. *Cibotium* is a tropical native medicinal plant in the Malaysian Peninsula and parts of China. It is an anti-inflammatory plant and is used in contradiction of rheumatic and menstruation problems, as well as herniated discs and hyperosteogeny [13, 14]. There are many phenolic compounds in *Cibotium* that are potent antioxidants and strong chelators. The rhizomes are comprised of approximately β-sitosterol, caffeic acid, daucosterol, alternariol, 5-hydroxymethyl-2-furancarboxaldehyde, (3R)-des-O-methyl lasiodiplodin, protocatechuic aldehyde, (24R)-stigmast-4-ene-3-one, onitin, 24-methylenecycloartanol, protocatechuic acid, n-butyl-β-d fructopyranoside, palmitic acid, 1-monopalmitin, d-glucose and 30% starch [15]. It has been confirmed that *C. barometz* obstructs osteoclast creation with no effects on cell viability [16]. The hairof *Cibotium* is a staple ingredient in the ointments that are applied in natural treatments, such as to stop bleeding [17]. The objective of our study was to evaluate the stomach-protective effect of *C. barometz* hair ethanol extracts on ethanol-induced stomach ulcers in rats.

RETRACTED

## Results

### Antiulcer study

#### Gross estimations

The results that pre-treated with *C. barometz* hair ethanol extract of male SD rats shown significant reduced of the ulcer area with compared to the ulcer groups (Table 1, Fig. 1) at four different doses in the pre-treated animals groups (62.5 mg\kg, 125 mg\kg, 250 mg\kg, 500 mg\kg) that were induced by ethanol 95%. However, the significant inhibition percentage of the ulcer area increased in rats pre-treated with *C. barometz* hair at doses of 62.5 mg\kg, 250 mg\kg, 125 mg\kg, and 500 mg\kg by 68.5%, 74.7%, 75.6%, and 78.5% respectively.

**Table 1:** Effect of the *C. barometz* hair extracts on the mucus weight, pH of stomach content, ulcer area, and % inhibition of ulcer area in the stomach

Animal groups	No group	Pre-treatment 5 ml/kg	Mucus weights (g)	PH (acidity)	Ulcer area (mm2)	Inhibition %
Normal control	G1	10% Tween20	2.28 ± 0.37^*^	7.16 ± 0.94^*^	-	-
Ulcer control	G2	10% Tween20	0.75 ± 0.37	2.76 ± 0.69	802.71 ± 87.32	-
Omeprazole	G3	20 mg/kg	1.92 ± 0.15^*^	5.71 ± 1.20^*^	95.71 ± 50.02^*^	88.1^*^
*C. barometz* hair extract	G4	(62.5 mg/kg)	1.86 ± 0.27^*^	4.27 ± 0.91^*^	253.20 ± 74.05^*^	68.5^*^
	G5	(125 mg/kg)	1.87 ± 0.12^*^	4.52 ± 1.15^*^	202.80 ± 32.01^*^	74.7^*^
	G6	(250 mg/kg)	2.00 ± 0.57^*^	5.12 ± 1.35^*^	195.60 ± 34.50^*^	75.6^*^
	G7	(500 mg/kg)	2.17 ± 0.51^*^	4.56 ± 1.26^*^	172.80 ± 53.10^*^	78.5^*^

^*^The values are expressed as the mean ± SEM. Indicates significance at *p < 0.05* compared to the ulcerated group

**Fig. 1:** The effect of *C. barometz* hair on the macroscopic appearance of the stomach mucosa in alcohol-induced stomach mucosal injuries in male SD rats. G1 (Normal control group) exhibited no injuries to the gastric mucosa, G2 (Ulcer control group) had severe injuries to the stomach mucosa, G3 (Omeprazole) showed mild disruptions of the surface epithelium in the gastric mucosa. G4 (62.5 mg/kg), G5 (125 mg/kg), G6 (250 mg/kg), G7 (500 mg/kg) doses of *C. barometz* hair extract had moderate to mild disruptions of the surface epithelium in the gastric mucosa in a dose-dependent manner. Black arrow points to the hemorrhagic bands

### Gastric mucus content and acidity

The outcomes that shown in Table 1, the ulcerated SD rat group produced the lowest gastric mucosa mucus content, while animal groups pre-treated with G7 (500 mg/kg) and G6 (250 mg/kg) of *C. barometz* hair exhibited significant increasing in the mucus weight (g) with respect to G2 (ulcer control rats). However, pre-treatment with *C. barometz* hair (G4 to G7) produced a significant increase in the pH of the stomach contents compared to the ulcer control rats (G2).

RETRACTED

### Histological protocol of evaluation the stomach injuries

#### Hematoxylin and eosin and Periodic Acid Schiff (PAS) stainings

Histology revealed comprehensive damage to the stomach mucosa in the ulcer control rats. Moreover, the ulcerated rat control group had necrotic lesions in the deep gastric mucosa that demonstrated extensive leucocyte infiltration and edema of the submucosal layer, as shown in Fig. 2. Conversely, the animals pre-fed with *C. barometz* hair extract in the G4 - G7 groups presented relatively enhanced protection of the stomach mucosa with a depression in or lack of infiltration of leucocytes and edema (Fig. 2). *C. barometz* hair extracts revealed defending effects in a dose-dependent manner and showed remarkably improved protection of the stomach epithelium. The gastric mucosa in the pre-treated experimental groups, depending on the dose, exhibited a gradual increase in PAS staining intensity, indicated by the accumulation of the magenta color in the mucosal cell layer compared to the ulcer control group (Fig. 3). Additionally, this magenta staining was reduced and was not plentiful in the gastric mucosa of the ulcer group where the ulcer was induced with ethanol.

**Fig. 2:** The effect of *C. barometz* on the histology (H and E staining) of ethanol-induced stomach mucosa damage in male SD rats. G1 (Normal control group) had intact surface mucosal epithelium with no lesions; G2 (Ulcer control group) had a severe distraction of the surface epithelium and necrotic lesions; G3 (Omeprazole) had a mild distraction of the surface epithelium and reduction in the submucosal edema with inflammatory cells infiltration. The animals pretreated with *C.* barometz extract in G4 (62.5 mg/kg), G5 (125 mg/kg), G6 (250 mg/kg) and G7 (500 mg/kg) groups revealed a moderate to mild disruption of the surface epithelium, a reduction in submucosal edema and inflammatory cells infiltration in a dose-dependent manner as shown by lowering in or absence of the ulcer area (white arrow), submucosal edema and inflammatory cells infiltration (blue arrow). (Scale bar = 100 μm)

**Fig. 3:** The effect of *C. barometz* on stomach tissue glycoprotein PAS staining in ethanol-induced gastric ulcers in SD male rats. G1 (Normal control group) had no accumulation of the magenta color in the mucosal cell layer; G2 (Ulcer control group) had decreased levels of the magenta color, G3 (Omeprazole), G4 (62.5 mg/kg), G5 (125 mg/kg), G6 (250 mg/kg), and G7 (500 mg/kg) showed increases in PAS staining intensity in mucosal cells layer compared to the ulcerated group, independent of dose. The red arrow indicates the PAS staining of glycoprotein. (Scale bar = 100 μm)

RETRACTED

### Immunohistochemistry

In the gastric mucosa, the expression of the HSP70 protein was down-regulated in the ulcerated group (G2), but significantly up-regulated in the animals pre-treated with omeprazole (G3) and with *C. barometz* hair extract (G4 to G7), as displayed in Fig. 4. Additionally, the immunohistochemical staining of the Bax proteins (Fig. 5) in the gastric mucosa revealed up-regulation in the ulcerated group while a significant down-regulation was demonstrated in rats pre-treated with *C. barometz* extract.

**Fig. 4:** Immunohistochemistry study of HSP70 expression in the stomach mucosa of SD male rats. G1 (Normal control group), G2 (Ulcer control group), G3 (Omeprazole), G4 (62.5 mg/kg), G5 (125 mg/kg), G6 (250 mg/kg) and G7 (500 mg/kg). HSP70 protein expression was up-regulated in animals pre-treated with C. barometz in a dose-dependent manner and HSP70 protein expression was also up-regulated with omeprazole. Down-regulation appeared in the ulcerated control group (Scale bar = 100 μm). All data are stated as the mean ± SEM. The mean difference was significant at the *P < 0.05* level compared to the normal control group

**Fig. 5:** Immunohistochemistry study of Bax expression the protein in the stomach mucosa of SD male rats. G1 (Normal control group), G2 (Ulcer control group), G3 (Omeprazole), G4 (62.5 mg/kg), G5 (125 mg/kg), G6 (250 mg/kg) and G7 (500 mg/kg). Bax protein expression was down-regulated in rats pre-treated with omeprazole and *C. barometz* in a dose-dependent manner. Bax was up-regulated in the ulcerated control group. (Scale bar = 100 μm). All data are stated as the mean ± SEM. The mean difference was significant at the *P < 0.05* level compared to the normal control group

### Measurement of antioxidant enzymes and membrane lipid peroxidation (MDA) of stomach

A significant reduction was observed in endogenous antioxidants enzymes (SOD, CAT and GPx) activities for the ulcer group of male SD rats. However, the rats pre-treated with *C. barometz* hair displayed an elevation of all antioxidant activities with respect to the (G2) ulcer group as shown in Figs. 6a, b, and c. The SOD enzyme activities were significantly higher at doses for G5 of *C. barometz* than G2 (Fig. 6a). The CAT enzyme activities illustrate the significant increases in G4, G5, G6 groups compared to G2 as shown in Fig. 6b. The GPx enzyme activities for gastric mucosal homogenates revealed significant increasing in the rats pre-fed with four doses of *C. barometz* hair ethanol extract with respect to G2 as shown in Fig. 6c. Additionally, the MDA level of *C. barometz* hair extract in G4, G5, G6 and G7 were significant lower than in the G2 ulcerated control group as seen in Fig. 6d.

RETRACTED

**Fig. 6:** Effect of *C. barometz* hair ethanol extracts on gastric tissue homogenate of superoxide dismutase (SOD), catalase (CAT), glutathione (GPx) and malondialdehyde (MDA) assays. G1 (Normal control group), G2 (Ulcer control group), G3 (Omeprazole), G4 (62.5 mg/kg), G5 (125 mg/kg), G6 (250 mg/kg) and G7 (500 mg/kg) of *C. barometz* hair ethanol extract. All values (in triplicate) are expressed as the mean ± SEM. * significant at *p* <0.05 compared to ulcerated group. SOD, CAT and GPx, antioxidant activities were higher in G1, G3 and G4 to G7 than in G2, although the MDA levels of G2 were higher than those of the other groups

### Acute toxicity test of *C. barometz* hair

All SD rats that were treated with *C. barometz* hair ethanol extract demonstrated no mortality and toxic signs in the experiment. There were no signs of hepatotoxic or nephrotoxic effects, which were evaluated histologically and biochemically (Fig. 7). Additionally, there were no body weight variations or abnormal physiological or behavioral changes at 2 g/kg and 5 g/kg doses during the 14 days, compared to the control group that was given 10% Tween 20.

**Fig. 7:** Histological slides of the liver and kidney sections for the acute toxicity experiment. Animals treated with 5 mL/kg of the vehicle (10% Tween 20) **a** and **b**. Animals treated with 2000 mg/kg (2 mL/kg) of the *C. barometz* hair extract **c** and **d**. Animals treated with 5000 mg/kg (5 mL/kg) of the *C. barometz* hair extract **e** and **f**. No significant changes were observed in the structures of the liver and kidney among the treated and control groups (hematoxylin and eosin stain; scale bar = 100 μm)

### Antioxidants activities of ethanol extract of *C. barometz* hair

#### Ferric reducing antioxidant power (FRAP) Test

*C. barometz* hair antioxidant activity in vitro was measured totally using the FRAP test. Fig. 8 revealed the decline of ferric to ferrous ions that indicated a higher FRAP value for *C. barometz* hair (756.0 ± 0.038 μmol Fe (II)/g) than BHT (261.0 ± 0.015 μmol Fe (II)/g) and ascorbic acid (457.7 ± 0.009 μmol Fe (II)/g). However, the value was less than for quercetin (1544.3 ± 0.021 μmol Fe (II)/g) and gallic acid (1774.3 ± 0.003 μmol Fe (II)/g) standards.

**Fig. 8:** FRAP test for total antioxidant activity evaluation of *C. barometz* hair extract with reference synthetic standards (BHT, ascorbic acid, quercetin, and gallic acid) were determined. All values are in triplicate and represented as the mean ± SEM

### The Scavenging of diphenyl - picrylhydrazyl radical activity (DPPH) test

*C. barometz* hair scavenging of DPPH free radicals was assessed using the DPPH test. Fig. 9 demonstrated the inhibition% of the DPPH free-radical scavenging activity of *C. barometz* hair that was 54.8% with an IC_50_ value of 45.6 ± 0.038 μg/mL. It was associated to the standards BHT, ascorbic acid, quercetin and gallic acid. The % inhibition of DPPH free-radicals scavenging activities of the standards was 51.63, 64.11, 87.52, and 55.47% with an IC_50_ value of 9.1 ± 0.01 μg/mL, 4.9 ± 0.02 μg/mL, 1.8 ± 0.001 μg/mL, 1.4 ± 0.02 μg/mL, respectively.

RETRACTED

**Fig. 9:** DPPH test for free radical scavenging activity (% inhibition) of *C. barometz* hair ethanol extract with reference synthetic standards (BHT, ascorbic acid, quercetin, and gallic acid). All values are in triplicate and represented as the mean ± SEM

## Discussion

Traditional medicine has become an important type of alternative medicine in many countries. Several medicinal plants have been used to protect the stomach from a number of ulcerative agents. One type of medicinal plant is *C. barometz* leaves, which are used to stop bleeding [13]. In this study, the results of acute toxicity experiment revealed no signs of toxicity or mortality in vivo and no variations in kidney and liver on biochemical investigation. Additionally, no differences in body weights were observed for both sex SD rats. These findings corroborate previous studies [18–20]. Our data suggest that *C. barometz* hair extract has high free-radicals scavengings and antioxidant activities in vitro. Our results agree with a previous report that indicated that the consumption of medicinal plants that contain natural antioxidants can reduce free radicals and protect biological molecules from oxidative injury [21]. *C. barometz* hair is one of the medicinal plants that have medicinal properties and natural antioxidants [17]. *C. barometz* hair displays good free-radical scavenging activity and ferric-decreasing antioxidant power in a Fe^3+^-dependent hydroxyl-radical generation assay [22]. This outcome agrees with earlier studies of *C. barometz*, in which it showed a greater antioxidant activity [23]. Our data indicate that significant protection of stomach wall mucosa and decreases in ulcer area are observed in rats pre-fed with *C. barometz* extract. Our observation is consistent with the findings of several other studies [4, 12, 24].

We also observed a significant elevation of stomach mucus content and pH in rats pre-fed with *C. barometz* hair extract compared to category of the ulcer control rats. This shows the extracted plant of *C. barometz* is able to protect the mucosal layer of the stomach from destructive causes. These results are similar to those previously reported by others [25–30]. A severe distraction of the gastric mucosa layer, edema and leucocyte penetration of submucosal layers were apparent in the ulcer control rats compared with rats pre-fed with *C. barometz* hair extract. The rats treated with *C. barometz* hair extract displayed a mild distraction of stomach epithelium and reduced edema and inflammatory cell penetration of the submucosal layers. Similarly, many studies have also observed mild distraction of stomach mucosa, mild edema and penetration of inflammatory cells in the submucosal layers [31–35]. Additionally, the condensing of the submucosal layer was detected in the ulcerated group where there was edema and hemorrhagic abrasions in the mucosal layer, which is an indicator of ethanol damage. Absolute ethanol harshly damages the stomach glandular epithelium leading to augmented neutrophils access into the disrupted stomach mucosa. The presence of oxygen free radicals resulting from the penetration of neutrophils in the wounded gastric wall can damage stomach gastric mucosa in rats [34, 36]. Neutrophils are the main sources of inflammatory mediators and can release the potent reactive oxygen species, which are cytotoxic and can promote tissue injury [37]. Furthermore, neutrophils that congregate in the stomach mucosa have been exposed to irritation through the microcirculatory defect [38]. The present study illustrated strong staining of glycoprotein discharge of stomach glandular epithelium in rats pre-fed with *C. barometz* extract. Mucus released from the stomach epithelium performs one of the vital mechanism of stomach mucosal barrier resistance against absolute ethanol [39, 40]. Mucus and bicarbonate liberation may have a considerable role in ulcer development because the mucus/bicarbonate layers guards newly produced cells from acidic and peptic damage [9, 41, 42]. The amplified production of mucus in the present work was an indicator of local mucosal defense in the stomach and can be described as the possible cytoprotective mechanism. Numerous studies have suggested that the gastroprotective defense is due to increased mucosal resistance, and a decline in aggressive factors, primarily acid and pepsin [43–45].

RETRACTED

The consequences of the present immunohistochemistry experiments indicate that rats pre-fed with *C. barometz* hair displayed an up-regulation of HSP70 proteins that contributed to the protection of stomach cells from heat shock, oxidative stress, and down-regulation of the Bax proteins. Earlier studies reported that there was up-regulation of HSP70 protein in animals fed with plant extracts [28, 34]. However, the down-regulation of Heat shock protein expression appeared in the ulcer control animals as a gastric injury marker. This is consistent with the results from other studies [20, 46]. Up-regulation of HSP70 protein in the stomach wall mucosa in animals pre-fed with *C. barometz* hair extract may stop the initiation of damage to the gastric epithelium upon exposure to absolute alcohol [23, 32]. The HSP70 protein protected mitochondria and delayed a stress-induced apoptotic programmer [47]. Our data suggest that Bax immune-staining confirmed that rats fed with *C. barometz* hair extract displayed increased an expression of the Bax protein. Thus, these results demonstrate that *C. barometz* hair extract is a protective agent and prevents alcohol-induced damage to the rat stomach, which is associated with decreased expression of the Bax protein. Similarly, many amendments have been described by many investigators [18, 48]. Animals pre-fed with *C. barometz* hair extract displayed decreased expression of the Bax protein. On the other hand, up-regulation of Bax was observed in the ulcer control group. Bax is a key protein that is linked to apoptosis during mitochondrial damage and plays a significant role in the disruption of stomach mucosal integrity that is observed after ethanol administration [11, 12].

The results from the present work demonstrated that rats pre-fed with *C. barometz* displayed an increase in the activity of endogenous antioxidant enzymes (SOD, GPx, CAT) and a decrease in MDA levels in the stomach compared to the ulcer control rats. These findings are consistent with observations from other studies [7, 32]. Therefore, the elevation of SOD and GPx enzymatic activities leads to increased scavenging of superoxides, hydrogen peroxide, hydroxyl and lipid peroxyl radicals, resulting in a reduction in tissue damage [9, 49]. Additionally, increases in CAT enzymatic antioxidant activity rapidly converted the peroxyl radicals into biologically safe substance, such as water [1]. In contrast, the low levels of MDA reduced lipid peroxidation and ROS (reactive oxygen species) which are products of oxidative gastric damage [8]. Taken together, our observations suggest that *C. barometz* hair facilitates gastric mucosa protection due to its scavenging of free radicals and anti-inflammatory effects [5, 6].

## Conclusion

Our study demonstrates that *C. barometz* hair has beneficial and dose-dependent anti-ulcer effects against ethanol-induced acute stomach hemorrhagic injuries in SD rats. The gastro-protective effects of this effective medicinal plant could be associated with free radicals scavenging activities, elevated levels of pH and gastric mucus glycoprotein, increases in the cellular endogenous enzymes activity of SOD, CAT and GPx antioxidants, and a reduction in MDA levels. Additionally, these effects may be due to HSP70 up-regulation and Bax protein down-regulation. Thus, *C. barometz* hair is a promising gastro-protective agent that can potentially be used to treat gastric ulcers.

RETRACTED

## Methods

### Plant extraction

*C. barometz* hair was identified and collected by the Herbarium of Rimba Ilmu, University of Malaya, Kuala Lumpur voucher No KLU 48648. One hundred grams of dried plants were soaked for five days in 900 ml of 95% ethanol and stirred daily in a laboratory glass bottle (1 L). Next, filter papers (Whatman No. 1) were used to filter the mixture and the ethanol (EtOH) extraction and distillation of *C. barometz* was accomplished under reduced pressures in a Buchi Rotary Evaporator R-215 (Chemoph-arm Sdn. Bhd., Switzerland). The *C. barometz* hair extract produced a 1.79% solution (dark-yellow; w/w). For acute toxicity, *C. barometz* extracst were diluted in 10% Tween 20 and administered to experimental rats orally at doses of 2 g/kg and 5 g/kg [50]. For anti-ulcer activity against ethanol-induced stomach mucosal damage, it was diluted in 10% Tween 20 at doses of 62.5, 125, 250, and 500 mg/kg body weight for oral administration as previously described [46].

### Gastric ulcer test

#### Omeprazole

Omeprazole was purchasdd from the University Malaya Medical Centre (UMMC) Pharmacy to use as a reference standard medication for gastric ulcers. For oral administration, omeprazole was dissolved in 10% Tween 20 and fed to animals at a dose of 20 mg/kg body weight (5 mL/kg) [18].

### Ethanol-induced gastric ulceration

The healthy adult male SD rats (181-208 g) were obtained from the Experimental Animal House, Faculty of Medicine at the University of Malaya. The animals were distributed into seven groups (*n* = 6 per group). Each animal was fasted for 24 h and fasted from water for 2 h prior to the experiment. The animals were housed in wire-bottomed cages to prevent coprophagy. Group 1 (vehicle group) and Group 2 (ulcer group) were orally administered 10% Tween 20 (5 mL/kg). Group 3 (reference control group) was fed 20 mg/kg of omeprazole orally. Groups 4, 5, 6 and 7 were orally administered the doses of 62.5, 125, 250, and 500 mg/kg of *C. barometz* hair extract, respectively. After one hour, Group 1 rats were administered 10% Tween 20 (5 mL/kg), and groups 2-7 rats were given the absolute alcohol (5 mL/kg) (Golbabapour et al.,[14]). Then, all animals were an overdose anesthetized using xylazine and ketamine (150 and 15 mg/kg), and after one hour, a cervical dislocation was performed for direct excision of their stomachs.

### Measurement of the stomach juice acidity and mucus contents

The stomach of each rat was untied alongside the greater curvature. The stomach contents were measured for the hydrogen ion concentrations using a pH meter titration with 0.1 N NaOH. The acid contents were expressed as meq/l. For each rat, the mucosa of stomach wasscraped slightly using the histological section slides, and the mucus in each stomach was weighed using the electronic balance [24].

RETRACTED

### Gross stomach injury evaluation

Ulcers of the stomach mucosa appeared as extended hemorrhagic bands of abrasions parallel to the long axis in the gut. In each gut, the length and width of ulcers (mm) were measured using the plan meter (10 × 10 mm^2^ = ulcer area) under a dissecting microscope (1.8x). The ulcer area was estimated by calculating number of the small squares, 2 mm × 2 mm, includingthe length and width of ulcer bands. For each stomach, the sum of the areas of all lesions was applied in the ulcer area (UA) calculations with the sum of small squares × 4 × 1.8 = UA (mm^2^), as previously reported by Rahim et al. [51]. The following equation in the calculation of theinhibition percentage was used in this study as previously described by Indran et al. [43]:

$$ \mathrm{Inhibition}\%=\left[\left(\mathrm{U}\mathrm{A}\mathrm{control}\hbox{-} {\textstyle}\mathrm{U}\mathrm{A}\mathrm{treated}\right)/\mathrm{U}\mathrm{A}\mathrm{control}\right]\times 100 $$

### Histological evaluation of stomach injuries

#### Hematoxylin and eosin staining

For each rat, the stomach wall specimens were put in 10% buffered formalin for fixation, processed in machine of tissue-processing (Leica, Germany) and paraffin-embedded. For histological assessments, slides of the stomach sections were prepared at a 5 μm thickness and stained with staining of hematoxylin and eosin (H and E) [52].

### Mucosal glycoprotein staining

To assess the mucus productions in the stomach, selected slides were put in the staining of Periodic Acid- Schiff (PAS), following the manufacturer’s instructions (Sigma Commercial Kits). The glandular portions of tissues were stained with this type of staining to visualize the production of mucus and changes in the basic and acidic glycoproteins. The light microscope (Nikon, Japan) was used to photograph then to observe any of the mucus produced (Nikon, Japan) [53].

### Immunohistochemistry staining

Animal Research Kit (ARKTM) was used to detect the immunohistochemical localization proteins of HSP70 (1:100) and Bax (1: 200) on the study slides. Both antibodies were bought from Santa Cruz Biotechnology, Inc., California, USA. Briefly, the slides of each tissue were put in a hot air oven (60^°^C) for 25 min (Venticell, MMM, Einrichtungen, Germany). Each tissue slides was de-paraffinized by xylene and re-hydrated by graded alcoholism solutions. The antigens retrieval were achieved using the microwave boiling of each samples in sodium citrate buffer (10 mM). After that, the endogenous peroxidase enzymes were blocked via hydrogen peroxide (0.03%) containing sodium azides then each tissue sections was put gently in the rinsing buffer. The slides were incubated with HSP70 (1: 100) or Bax (1: 200) biotinylated first antibodies for 15 min. Next, they were rinsed with the rinse buffer to put them in the buffer bath. Each slide was kept in the humidified chambers. For 15 min, the sections of immunohistochemistry slides were incubated through streptavidin conjugated to horseradish peroxidase in PBS containing an anti-microbial agent (streptavidin–HRP). They were put again in the rinsing buffer then in the buffer bath before incubation with diaminobenzidine substrates chromagen for 5 min. the slides of this experiment were washed, counterstained with hematoxylin (5 s), dipped in 0.037 M/L of weak ammonia for 10 times. The washing through distilled water is important before the mounting of the slides with cover slips. Affirmative identification of this immunostaining was observed in the brown coloration of tissue sections under the light microscope. Protein expression levels were quantitated by the NIH image J software programs. The data are shown by mean ± SD and statistical significance was expressed as *P < 0.05*.

RETRACTED

### Antioxidants activity of gastric homogenate

#### Preparations of stomach homogenates

For each stomach tissue, the samples were washed comprehensively by the ice-cold potassium buffer phosphate (PBS). Each stomach homogenates (10% (w/v) was prepared with the ice-cold 50 mM (PBS) (pH 7.4) using the tissue homogenizer (Polytron, Heidolph RZR 1, Germany). They were centrifuged for 15 min at 10,000 rpm (4 ^*°*^C) using refrigerated centrifuge Rotofix 32 (Hettich Zentrifugen, Germany). Next, the supernatants were used for the evaluation of antioxidants activity and lipid peroxidation levels.

### Evaluation of antioxidant activities of gastric homogenate

The commercial kits of Cayman Chemical Company, Ann Arbor, USA were purchased for assessment the SOD, CAT and GPx activities of the stomach tissues. The manufacturer’s procedures were used for the determination of antioxidants activities in the gastric tissue supernatants of each sample.

### Measurements of lipid peroxidation (MDA) levels of stomach homogenates

Lipoperoxidation of the mucus membrane in the gastric epithelium was determined by purchasing the commercial kit from (Cayman Chemical Company, Ann Arbor, USA.

RETRACTED

### Antioxidant activity in vitro

#### Ferric-reducing antioxidant power (FRAP) assessment

In brief, FRAP reagents were used using freshly preparing from acetate buffer (pH 3.6), 10 mM TPTZ [2,4,6-Tri(2-pyridyl)- s-triazine] solution in HCl (40 mM), and 20 mM Fe (III) chloride solution in proportions of 10:1:1 (v/v), correspondingly. Butylated hydroxytoluene (BHT), ascorbic acid, quercetin, and gallic acid were used as controls of the test. Ten microliters of each plant extract, standard and controls were put into 300 μL of the FRAP reagent (in triplicate) and left in a dark place for 4 min. Then the absorbance was recorded at 593 nm via a power wave × 340 ELISA Reader (Bio-Tek Instruments, Inc., Winooski, VT, USA). The standard curve was constructed linearly (R2 = 0.998) between 100 and 1000 M FeSO_4_. The outcomes were expressed as M Fe (II)/g dry weight of the extract.

### Scavenging of diphenyl-picrylhydrazyl radical activity (DPPH) assay

A stock solution (1 mg/1 mL) of the extracted medicinal plant was prepared then diluted to produce five different concentrations (50, 25, 12.5, 6.25, 3.125, 1.56 μg/mL), and the antioxidant ascorbic acid was used as the standard. 5 μL of *C. baromtz* and standard were mixed with 195 μL DPPH (40× dilution) in triplicate. After that, each mixture was incubated at 37^°^C. The absorbance value was measured for 2 h at 20 min intervals using a spectrophotometer of power wave × 340 on the ELISA Reader (Bio-Tek Instruments, Inc., Winooski, VT, USA) at 515 nm.

The radical scavenging activity was estimated using this formula:

$$ \%\ \mathrm{inhibition} = \left\{\left(\mathrm{AB}\hbox{--} \mathrm{AA}\right)/\mathrm{AB}\right\}\times 100 $$

AB is the absorption of the blank sample; AA is the absorption of the tested samples. The inhibitory concentration 50% was determined besides the kinetics of scavenging reactions of DPPH. BHT, ascorbic acid, quercetin, and gallic acid were also verified against DPPH as positive controls [22].

### Acute toxicity and experimental SD rats

Adult Sprague Dawley rats (male and female, 6–8 weeks old), were attained from the Animal House, Faculty of Medicine, University of Malaya, Kuala Lumpur (Ethic no.PM/30/05/2012/NSIAW (R). The body weight of the rats was between 166–190 g. Each rat was fed standard animal pellets and tap water. The acute toxicity test was performed to determine the nontoxic dose of *C. barometz* hair. Thirty six SD rats (18 males and 18 females) were randomly separated equally into three categories each labeled as vehicle (10% Tween 20), 2 g/kg, and 5 g/kg of *C. barometz* hair preparation [25, 50, 54, 55]. The animals were fasted overnight before dosing (food but not water), and then the diet was withdrawn for an additional three to four hours after dosing. SD rats were observed for 30 min and 2, 4, 8, 24 and 48 h after feeding at the beginning of toxicological assessments. Mortality was documented over a period of 14 days. On the 15^th^ day, the animals were injected with an overdose of anesthesia (xylazine with ketamine) then blood, kidneys and liver were obtained. Histology and serum biochemical parameters were assessed according to the OECD guidelines [56].

RETRACTED

### Statistical analysis

The statistically significant differences among the groups were measured by the SPSS statistical program software version 20. A one-way analysis of variance (ANOVA) was used with Tukey’s multiple comparison post hoc test. All data were reported as the mean ± SEM. A value of *P < 0.05* was reflected significant.
